# A Reparameterization Multifeature Fusion CNN for Arrhythmia Heartbeats Classification

**DOI:** 10.1155/2022/7401175

**Published:** 2022-11-23

**Authors:** Dengyong Zhang, Haoting Zhou, Feng Li, Lebing Zhang, Jianxin Wang

**Affiliations:** ^1^Hunan Provincial Key Laboratory of Intelligent Processing of Big Data on Transportation, Changsha University of Science and Technology, Changsha 410114, China; ^2^School of Computer and Communication Engineering, Changsha University of Science and Technology, Changsha 410114, China; ^3^Huaihua University, Huaihua 418000, China

## Abstract

Aiming at arrhythmia heartbeats classification, a novel multifeature fusion deep learning-based method is proposed. The stationary wavelet transforms (SWT) and RR interval features are firstly extracted. Based on the traditional one-dimensional convolutional neural network (1D-CNN), a parallel multibranch convolutional network is designed for training. The subband of SWT is input into the multiscale 1D-CNN separately. The output fused with RR interval features are fed to the fully connected layer for classification. To achieve the lightweight network while maintaining the powerful inference capability of the multibranch structure, the redundant branches of the network are removed by reparameterization. Experimental results and analysis show that it outperforms existing methods by many in arrhythmic heartbeat classification.

## 1. Introduction

The heart is a muscle that contracts in a rhythmic way to pump blood throughout the body. The activity of the heart generates electric currents on the surface of the body, which cause changes in the electrical potential of the skin [1]. Electrocardiograph (ECG), a medical technology widely used in clinical medicine, can noninvasively detects the electrical potential changes on the skin caused by cardiac activity. Doctors can diagnose cardiovascular diseases by observing the ECG. However, only relying on doctors to analyze ECG is not only inefficient but also prone to visual fatigue when working for long hours. To reduce the burden on doctors, the computer aided diagnosis (CAD) system is a reliable solution. It utilize machine learning (ML) or deep learning (DL) methods to diagnose cardiovascular diseases by monitoring ECGs, which can help doctors determine the right treatment plan and save valuable treatment time. Therefore, the automatic classification system of electrocardiogram is of great significance to improve medical efficiency, reduce medical cost and prevent heart disease [2].

The arrhythmia heartbeats classification work is mainly divided into four stages: preprocessing, heartbeat segmentation, feature extraction, and classification. The main work of preprocessing is to denoise the ECG signal to improve the signal-to-noise ratio (SNR). Common methods such as wavelet transform (WT) [3], empirical mode decomposition (EMD) [4], and denoising autoencoder [5]. The heartbeat segmentation is used to get the segmentation reference points of the ECG recording to facilitate the subsequent signal processing, through detected R peaks or QRS complexes [1]. In the feature extraction step, some useful features related to arrhythmia heartbeats are extracted from ECGs, such as RR intervals [6], wavelets [7], and local binary pattern (LBP) [8]. In the classification stage, the result of arrhythmia heartbeats can be identified by the ML and DL algorithm. For the ML algorithm, the classification results usually depend on whether the extracted features are accurate and suitable. While the DL algorithm is different, it can automatically extract abstract features from the input data and has stronger generalization than ML algorithms. Our proposed scheme fused multifeatures and reparameterized the designed parallel multibranch convolutional network. It is not only has a lightweight architecture but also achieves comparable performance to other DL methods. The main contributions of this paper are as follows.

- A multifeature fusion method for arrhythmia heartbeats classification was proposed. The SWT feature reflects the characteristics of the time and frequency domains, and the RR interval feature relates a single beat to other surrounding beats. The combination of SWT and RR interval features can effectively improve classification performance
- The reparameterization technology was utilized to lightweight the designed multibranch convolutional neural network structure. It maintains the model classification ability and eliminates the disadvantage of the high computational cost of the multibranch
- Experimental results and analysis illustrate the proposed method can achieve good performance. The average overall accuracy is 99.43% while keeping the designed network lightweight

The rest of the paper is organized as follows: the related works are introduced in Section 2. The proposed arrhythmia heartbeats classification scheme is described in Section 3. Experimental results and analysis are provided in Section 4. Finally, some conclusions are drawn in Section 5.

## 2. Related Work

Some researchers used traditional ML-based methods to realize arrhythmia heartbeats classification. Mondéjar-Guerra et al. [8] extracted wavelets, LBP, higher-order statistics (HOS), and their Morphological Descriptor features from denoised signals and obtained the classification results by support vector machines (SVMs). Tuncer et al. [9] used neighborhood component analysis (NCA) to reduce the dimensionality of extracted discrete wavelet transform (DWT) and 1-dimensional hexadecimal local pattern (1D-HBP) features, and used the K-nearest neighbor classification algorithm (KNN) for classification. Jha et al. [10] classify the arrhythmia heartbeats by tunable Q-wavelet transform (TQWT) from denoised the ECG signals.

In recent years, DL has been booming and involved in several fields, such as object detection [11], natural language processing [12], and image restoration [13]. In the field of heartbeat classification, more and more works are using DL algorithms. It also exhibits a strong ability to classify heartbeats. Mousavi and Afghah [14] used a synthetic minority oversampling technique (SMOTE) to solve the problem of sample imbalance, and then used a sequence-to-sequence with CNN model for classification. Yildirim et al. [15, 16] directly fed 10 s-long ECG segments into a 16-layer deep convolutional neural network to complete the classification efficiently. After that, they classified the original and compressed signals by long short-term memory (LSTM) network. The classification accuracy is 99.23% and 99.11%, respectively. Oh et al. [17] combined CNN and LSTM for heartbeats classification. Kiranyaz et al. [18] used 1D-CNN for heartbeats classification with good performance and low computational cost.

Furthermore, some researchers combined the traditional feature extraction method used in ML and DL methods for heartbeats classification. The traditional features reflected the differences between different categories of heartbeats, which can facilitate the DL model learning meaningfully semantic features. Shoughi and Dowlatshahi [19] used DWT and SMOTE oversampling algorithms for preprocessing and fed them into CNN and BLSTM networks. Nurmaini et al. [20] used stacked denoising autoencoders (DAEs), autoencoders (AEs), and deep neural networks (DNNs) for feature extraction and classification. El Bouny et al. [21] fed the original ECG signals and the extracted SWT features into a multiscale 1D-CNN, and the overall accuracy is 99.11%. Subsequently, they [22] used more SWT wavelet subbands, the maximum and connection schemes are used to fuse the output of multiscale 1D-CNN, and the overall accuracy rises to 99.58%. Ullah et al. [23] extracted Fourier features and input them into a CNN networks. Jun et al. [24] directly transformed the one-dimensional ECG signal into a two-dimensional image and used CNN to classify them. Allam et al. [25] used Stockwell transform and 2-dimensional residual network (2D-ResNet). Training the model with a small dataset achieves good classification results with good generalization. Rajput et al. [26] performed wavelet and short-time Fourier transform on the preprocessed signal and used dense neural network for classification. Liu et al. [27] used wavelet scattering transform and extracted time windows, which were downscaled and fed into a neural network, probabilistic neural network, and KNN classifiers for classification, respectively. Wang et al. [28] used CNN to extract features from the continuous wavelet transform signal of ECGs, and combined it with the RR interval features to classify the heartbeat by the fully connected layers. The classification results on supraventricular ectopic beats and ventricular ectopic beats outperform many existing schemes. Although the current DL-based heartbeats classification method can achieve good performance, their models have a huge number of parameters. It is not convenient to deploy these models on ECG machines with small storage space and slow computation speed.

To maintain a lightweight model, we first designed an original CNN-based heartbeats classification model. It fused the RR interval features and a multiscale 1D-CNN to extract features of three subbands of SWT. And then, the parallel convolutional layers are fused into a single convolutional layer by a reparameterization technique, which can greatly reduce the model's parameters.

## 3. Proposed Method

The proposed heartbeat classification framework contains four parts: SWT feature extraction module, RR interval feature extraction module, multibranch CNN module, and classifier module. For an input ECG signal, the SWT feature and RR interval feature are first extracted. After that, three subbands of SWT are fed to the multibranch CNN, which consisted of three reparameterization multiscale 1D-CNNs. Finally, the fusion features are used as the input of a multidense layer classifier, and then the 5 types of heartbeats are classified. The framework of the proposed scheme is shown in Figure 1.

### 3.1. SWT Feature Extraction

Wavelet transform is a commonly used transform in the field of ECG signal processing. It has an excellent ability to analyze nonstationary signals. For example, DWT [3, 8] is often used in the preprocessing and feature extraction stages, while it does not have the characteristics of transformation invariance. Therefore, we transfer to another wavelet transform, namely SWT. Same as DWT, SWT feeds the signal into a series of low-pass and high-pass filters, but instead of filtered downsampling, upsampling is implemented by zero-interpolation [29]. The low-pass filter gives the approximate coefficients and the high-pass filter gives the detail coefficients. The wavelet coefficients of the *j*^th^ level can be expressed as

(1) $$\begin{array}{c} D_{j}=H_{j}*A_{j-1},\\ A_{j}=L_{j}*A_{j-1}, \end{array}$$

where *H*_*j*_ and *L*_*j*_ represent the *j*^th^ stage high-pass and low-pass filters, and *D*_*j*_ and *A*_*j*_ represent the detail and approximation coefficients of the *j*^th^ stage. The 5-level SWT decomposition process is shown in Figure 2.

In this work, we used a five-level SWT and wavelet “db1” with a 1 × 2 filter.  Table 1 shows the frequency range of the five-level SWT subbands on the data sampled at 360 Hz in the MIT-BIH arrhythmia database while the main energy of the ECG signal is mainly concentrated in the frequency range of 3–40 Hz [30]. Therefore, the main energy of the ECG signal is contained in *D*_3_, *D*_4_, *D*_5_, and *A*_5_. Although the *A*_5_ subband has the signal energy of the ECG, the baseline wander noise is also in it. Considering that the network is as lightweight as possible, it is discarded. Therefore, only three subbands of SWT (*D*_3_, *D*_4_, and *D*_5_) are considered in our proposed scheme. The detail coefficients of *D*_3_, *D*_4_, and *D*_5_ obtained by *S* class ECG segments SWT were shown in Figure 3.

### 3.2. RR Interval Feature Extraction

Considering the significant difference in the heartbeat intervals of arrhythmias compared to normal ones, the RR interval features are also taken into account in our scheme. Inspired by previous work [26], four RR interval features were considered. There are previous-RR, post-RR, ratio-RR, and local-RR features. Previous-RR is the *R* peak interval between the current heartbeat and the previous heartbeat. Post-RR is the interval between the current heartbeat and the next heartbeat, and ratio-RR is the ratio of the pre-RR to the post-RR. The local-RR is the average of the ten previous-RR before the current heartbeat. To eliminate differences between patients, the mean *R* peak interval was subtracted from previous-RR, post-RR, and local-RR.

### 3.3. Multiscale 1D-CNN Reparameterization

Inspired by RepVGG [31], we use parallel convolutional layers (Conv1D) to form a multiscale feature of SWT to improve the classification effect.  Figure 4 shows the original network structure of the multiscale 1D-CNN without reparameterization in Figure 1. In this part, we will describe the detail of reparameterization multiscale 1D-CNN.

The Conv1d and batch normalized layer (BN) can be formula expressed as

(2) $$\begin{array}{c} \text{Conv}\left(x\right)=W\left(x\right)+b,\\ \text{BN}\left(x\right)=\gamma \frac{\left(x-\mu \right)}{\sigma }+\beta , \end{array}$$

where *x* is the input, *W*(*x*) is the convolution operation, *b* and *β* are the biases of the Conv1D and BN layers, respectively. And *μ*, *σ*, and *γ* are the mean, standard deviation, and learnable scale factors, respectively. The output of the Conv1D is used as the input of the BN to obtain as

(3) $$\begin{array}{c} \text{BN}\left(\text{Conv}\left(x\right)\right)=\gamma \frac{W\left(x\right)}{\sigma }+\gamma \frac{\left(b-\mu \right)}{\sigma }+\beta . \end{array}$$

The above formula can be regarded as a new Conv1D formula. Thus the Conv1D after fusion with the BN layer is formulated as follows:

(4) $$\begin{array}{c} \text{Con}{\text{v}}^{\prime }\left(x\right)=W^{\text{'}}\left(x\right)+b^{\prime }. \end{array}$$

where *W*′ = *γ*(*W*/*σ*), *b*′ = *γ*((*b* − *μ*)/*σ*) + *β*.Taking the first layer of multiscale 1D-CNN as an example, the reparameterization process is shown in Figure 4. Starting from the original two-scale structure, each Conv1D first needs to adsorb its BN separately, and the new Conv1D obtained is shown in Eq. (4). Then the 1 × 5 convolutional kernel is directly converted to 1 × 7 size by a zero-padding operation. Finally, the convolutional kernel parameter matrix and bias of the two Conv1D are directly added separately to obtain the merged convolutional layer. Therefore, two Conv1Ds and their BNs layers are fused to a new Conv1D.

In Figure 5, the 1 × 7 and 1 × 5 Conv1D have the same step, and the padding parameter of the latter is set to 1 while the former is set to 0 to ensure that the output tensor size of both is the same. Theoretically, any number of Conv1Ds can be fused, provided that the following conditions are satisfied: same step size; the kernel size of each Conv1D differs by a multiple of 2. By setting the padding of each Conv1D, it is ensured that the size of the tensor obtained after convolution of each Conv1D is the same. The fused network has fewer parameters than the original network and does not degrade the inference accuracy.

## 4. Experimental Results

In this part, the experimental datasets and evaluation criteria are first introduced, and then a series of experiments and analysis is used to illustrate the effectiveness of the proposed arrhythmia heartbeats classification scheme.

### 4.1. Dataset Setup

The MIT-BIH arrhythmia database [32] is a classic and excellent dataset in the field of ECG signal processing, and many studies on cardiac beat classification are based on this dataset. The dataset has been in an updated state since its creation. The MIT-BIH consists of 48 records from 47 different patients with a sampling frequency of 360*HZ*. We used the modified-lead II (MLII) in the dataset as the original signal. According to the classification standard of arrhythmia beats suggested by the American association of medical instrumentation (AAMI) standard [33], five heartbeats (normal, supraventricular ectopic beats, ventricular ectopic beats, fusion, and unknown beats) are classified. Noting that the annotation file in the MIT-BIH dataset [32] contains the information on QRS peak occurrence time and heartbeat type, and we take 99 samples and 156 samples on the left and right sides of the *R* peak, respectively. Thus, a heartbeat sample of length 256 was obtained (5-level SWT requires an input sample length of 2^n^, *n* > 5). The heartbeat segment is standardized by Z-score regularization, which is beneficial to the training of the model. Finally, 109398 heartbeats were extracted from MIT-BIH dataset, of which there are 90548 in normal class (*N*), 2779 in supraventricular ectopic beats (*S*) class, 7234 in ventricular ectopic beats (*V*) class, 802 in fusion (*F*) class, and 8035 in unknown beats (*Q*) class.

### 4.2. Evaluation Criteria

To evaluate the experimental results, four metrics: the sensitivity (Se), the specificity (Sp), the positive predictivity (P+), and the accuracy (Acc), are implemented for the performance analysis.

(5) $$\begin{array}{c} \text{Se}=\frac{\text{TP}}{\text{TP}+\text{FN}},\\ \text{Sp}=\frac{\text{TN}}{\text{TN}+\text{FP}},\\ \text{P}+=\frac{\text{TP}}{\text{TP}+\text{FP}},\\ \text{Acc}=\frac{\text{TP}+\text{TN}}{\text{TP}+\text{TN}+\text{FP}+\text{FN}}, \end{array}$$

where TP, FP, TN, and FN are the true positive, false positive, true negative, and false negative, respectively. In addition to this, the overall accuracy is used for evaluating the overall performance, it defined as

(6) $$\begin{array}{c} \text{Overall Acc}\left(\%\right)=\frac{\text{Total number of correctly classified}}{\text{Total number of heartbeats}}\times 100\%. \end{array}$$

### 4.3. Implementation Detail

In order to ensure the generalizability of the model and find the proper hyperparameters, the extracted 109,398 heartbeats are used for 10-fold cross-validation based on heartbeat-orientation. 10-fold cross-validation is used. The checkpoint technique from the skorch [34] library is utilized in the training to save the best model.

The proposed network uses cross-entropy loss function and Adam optimizer. The learning rate is empirically set as 0.001and the reduction is 0.1 per 12 epochs. The dropout rate is set as 10%. The stride of Conv1D is set as 1. The number of 1D-CNN convolutional kernels in the 3 layers is 8, 16, and 32, respectively. The kernel size and step size of the pooling layer are set as 3.

### 4.4. Original Multiscale 1D-CNN Structure Selection

To keep the original multiscale 1D-CNN lightweight, the classical 3-layer structure is taken into account. In order to find the most appropriate number of convolutional layers per layer for multiscale 1D-CNN, we did comparison experiments. In the first layer, a 1 × 7 Conv1D is fixed, and 1 × 5 and 1 × 3 Conv1D can be parallelized. The second and third layers are fixed with a 1 × 5 and 1 × 4 Conv1D, respectively. The corresponding layers can be paralleled with a 1 × 3 and 1 × 2 Conv1D, respectively. Here, four cases were taken into account, and 10-fold cross-validation technology was used to evaluate each case. The obtained average overall accuracy results are shown in Table 2. It can be found that the accuracy of case 3 achieves the best overall accuracy 99.43%, which is our proposed multiscale 1D-CNN structure before re-parameterization (as shown in Figure 5).

### 4.5. Performance Evaluation

By comparing the results of the proposed reparameterization network with the original ones, we find that the overall accuracy obtained by the two inferences is the same in the first 16 decimal places. It can be considered that the reparameterization will not affect the model inference results. The classification accuracy of five types of heartbeats is shown in Table 3. The proposed scheme achieves good average accuracy on different evaluation metrics. The average Se, Sp, P+, and Acc is 95.32%, 99.61%, 96.91%, and 99.77%, respectively. Furthermore, the confusion matrix obtained by 10-fold cross-validation is shown in Table 4. It can be found that the proposed scheme is good at distinguishing each heartbeats class (*S*, *V*, *F*, and *Q* classes), especially for the *Q* class.

Here, we show the overall accuracy, Se, and P+ of each fold classification during the 10-fold cross-validation, as shown in Figure 6. The average overall accuracy obtained is 99.43%. In the 9^rd^ fold, the best performance 99.52% can be achieved. Meanwhile, Se and P+ had the best results of 98.09% and 96.24% and appeared in the 5^th^ and 8^th^ folds. It can be found that the overall accuracy does not fluctuate too much during the 10-fold cross-validation. The results illustrate that the proposed scheme is stable and robust.

### 4.6. Performance Comparison

In order to evaluate the effectiveness of the proposed scheme, the performance comparison between the proposed method and some state- of-the-art arrhythmia heartbeat classification methods are listed in Tables 5. For fair comparison, all the compared methods are based on the MIT-BIH arrhythmia database. As seen from Table 5, the proposed method which used a simple 3 layers 1D-CNN network is able to achieve a comparable performance with other complex DL methods.

Furthermore, we conducted experiments using the patient-oriented dataset partitioning method proposed by de Chazal et al. [35] and obtained an overall accuracy of 96.14% in the DS2 dataset.

### 4.7. The Lightweight Brought by Reparameterization

To evaluate the effectiveness of reparameterization on lightweight, the third-party library thop is utilized. The number of parameters of the original multibranch CNN is 53989. After the reparameterization operation, the number of parameters decreased to 25301, which is 55.5% less than the original ones. For the floating-point operations (FLOPs), the original multibranch CNN is 85780800 and the FLOPs of the reparameterized multibranch CNN is 63273600, which is reduced by 26.24%. Combined with the accuracy after the reparameterization (see Section 4.5), it can be found that the reparameterization multibranch CNN can greatly reduce the computational cost without loss much on the inference results.

## 5. Conclusion

In this paper, a novel arrhythmia heartbeat classification scheme is proposed. Multifeature feature fusion-based method is first taken into account. The SWT subband feature and RR interval feature work together for improving the classification accuracy. The newly designed reparameterization multibranch CNN structure achieves a lightweight network while maintaining high heartbeat classification accuracy. The proposed scheme is evaluated on the MIT-BIH arrhythmia database and the average overall accuracy is 99.43%. Our future work will be focused on solving the problem of minority heartbeats classes being misclassified to *N* class.

## Figures and Tables

**Figure 1:** The overview of proposed automatic heartbeat classification scheme, 1 × 256 and 32 × 8 represent the input and output sizes of the multiscale 1D-CNN.

**Figure 2:** the 5-level SWT process.

**Figure 3:** Three detail coefficients *D*_3_, *D*_4_, and *D_5_* of decomposed ECG segments using SWT for class *S.*

**Figure 4:** Multi-scale 1D-CNN structure.

**Figure 5:** the reparameterization process, from left to right, is as follows: original structure; the fusion of Conv1D and BN layers; zero-filling of 1 × 5 kernels into 1 × 7 kernels; completion of the fusion.

**Figure 6:** The overall accuracy, Se, and P+ in each fold.

**Table 1:** The frequency range of 5-level SWT subbands.

SWT subband	Frequency range(Hz)
*D*_1_	90-180
*D*_2_	45-90
*D*_3_	22.5-45
*D*_4_	11.25-22.5
*D*_5_	5.625-11.25
*A*_5_	0-5.625

**Table 2:** Average overall accuracy obtained by ten-fold cross validation for each structure.

Case	The number of Conv1D in different layers (*x*_1_ − *x*_2_ − *x*_3_)	Overall Acc
1	1-1-1	99.37%
2	3-2-1	99.41%
3	3-2-2	99.41%
4	2-2-1 (proposed)	99.43%

*x*_1_ − *x*_2_ − *x*_3_, *x*_1_, *x*_2_, *x*_3_ represent the number of Conv1D in the first, second, and third layer, respectively.

**Table 3:** The classification accuracy for each heartbeat class.

	*N*	*S*	*V*	*F*	*Q*	Average
Se	99.78%	93.89%	98.51%	84.38%	99.68%	95.78%
Sp	98.34%	99.91%	99.88%	99.94%	99.98%	99.61%
P+	99.66%	96.31%	98.36%	90.97%	99.71%	96.98%
Acc	99.53%	99.75%	99.77%	99.79%	99.96%	99.77%

**Table 4:** Confusion matrix for five types of heartbeat classification results.

		*Predicted label*				
		*N*	*S*	*V*	*F*	*Q*
*True label*	*N*	90352	87	53	36	22
	*S*	142	2610	26	2	0
	*V*	68	10	7122	29	1
	*F*	77	3	45	675	0
	*Q*	24	0	2	0	8014

**Table 5:** Performance comparison with existing DL methods.

Authors	# heartbeats	# categories	Overall accuracy
El Bouny et al. [21]	109428	5	99.11%
Khalil and Adib [22]	45000	6	99.57%
Shoughi et al. [19]	113131	5	98.71%
Yildirim et al. [16]	100022	5	99.23%
Proposed method	109398	5	99.43%

## Data Availability

The software code and data used to support the findings of this study are available from the corresponding author upon request.
